# A Zinc Morpholine Complex Prevents HCl/Ethanol-Induced Gastric Ulcers in a Rat Model

**DOI:** 10.1038/srep29646

**Published:** 2016-07-27

**Authors:** Suzy M. Salama, Nura Suleiman Gwaram, Ahmed S. AlRashdi, Shaden A. M. Khalifa, Mahmood A. Abdulla, Hapipah M. Ali, Hesham R. El-Seedi

**Affiliations:** 1 Department of Biomedical Science, Faculty of Medicine, University of Malaya, 50603 Kuala Lumpur, Malaysia; 2 Department of Chemistry, Faculty of Science, University of Malaya, 50603 Kuala Lumpur, Malaysia; 3 Department of Experimental Hematology, Karolinska University Hospital, SE-141 86 Stockholm, Sweden; 4 Department of Molecular Biosciences, The Wenner-Gren Institute, Stockholm University, S-106 91 Stockholm, Sweden; 5 Department of Otolaryngology-Head and Neck Surgery Kumamoto University 1-1-1 Honjo, Kumamoto, Japan; 6 Division of Pharmacognosy, Department of Medicinal Chemistry, Uppsala University, Box 574, SE-75 123, Uppsala, Sweden

## Abstract

Zinc is a naturally occurring element with roles in wound healing and rescuing tissue integrity, particularly in the gastrointestinal system, where it can be detected in the mucosal and submucosal layers. Zinc chelates are known to have beneficial effects on the gastrointestinal mucosa and in cases of gastric ulcer. We synthesized complexes of zinc featuring a heterocyclic amine binding amino acids then investigated their ability to enhance the gastric self-repair. Zinc-morpholine complex, Zn(L)SCN, namely showed strong free-radical scavenging, promotion of the DNA and RNA polymerases reconstruction and suppression of cell damage. The complex’s mode of action is proposed to involve hydrogen bond formation via its bis(thiocyanato-k)zinc moiety. Zn(L)SCN complex had potent effects on gastric enzymatic activity both *in vitro* and *in vivo*. The complex disrupted the ulcerative process as demonstrated by changes in the intermediate metabolites of the oxidative pathway – specifically, reduction in the MDA levels and elevation of reduced glutathione together with an attenuation of oxidative DNA damage. Additionally, Zn(L)SCN restored the gastric mucosa, inhibited the production of pro-inflammatory cytokines (IL-6, TNF and the caspases), and preserved the gastric mucous balance. Zn(L)SCN thus exhibited anti-oxidative, anti-inflammatory and anti-apoptotic activities, all of which have cytoprotective effects on the gastric lining.

Human health and longevity are closely linked to the balance of the digestive system. Gastric ulcer and oesophageal reflux have common symptoms including nausea, heart burn and discomfort that affect the overall quality of life^1^. In recent years the link between modern lifestyles and digestive system disorders has been recognized. While no direct connection has yet been established between modern sedentary lifestyles and dietary habits (such as smoking, coffee consumption, eating fast food, and stress) and the symptoms of gastroesophageal reflux, there is evidence that fast food consumption worsens gastrointestinal performance and aggravates ulcers^2^. The best way to solve such stomach problems is arguably to find ways of restoring gastric homeostasis rather than simply providing medications to address their symptoms.

The secretion of gastric acid and digestive enzymes (pepsin, rennin, and lipases) is tightly regulated in healthy individuals. The gastric acid sterilizes the stomach’s contents and establishes a suitable environment for the activity of the secreted enzymes^3^, while mucus and digestive enzymes are secreted in a controlled manner to ensure that the stomach is protected from its highly acidic contents and that its contents retain sufficient enzymatic activity to support digestion. For optimal digestion, food should reside in the stomach for approximately an hour, which is sufficient for pre-digestion and for the gastric reflexes to stimulate the secretion of gastric acids and pepsin^4^. Other active enzymes derived from foods such as meat, vegetables, and fruits may also be present in the stomach. However, in individuals whose diet does not include foods that provide such enzymes on a regular basis, the entire sequence of the digestive process can become compromised. Fast, processed and overcooked foods lack essential digestive enzymes^5^, so their consumption forces the stomach to produce fluctuating amounts of acid in an attempt to compensate, which adversely affects the response of the gastroesophageal reflexes and creates a situation that allows aggressive bacteria such as *Helicobacter pylori* to thrive in the stomach. *H. pylori* and long-term usage of non-steroidal anti-inflammatory drugs (NSAIDs) are amongst the most common causes of gastric ulcer^6^. NSAIDs have soothing effects on the gastric receptors, inhibiting the production of prostaglandins which are important in protecting the stomach lining. This in turn makes the stomach more sensitive to excessive consumption of coffee and cigarettes, whose chemical constituents irritate the stomach in a way that is exacerbated by preexisting weaknesses of the gastroesophageal sphincter. This irritation induces gastric acid hypersecretion, increases in stress hormone levels, and suppression of the immune system^7^. Coffee and smoking are linked to several predisposing factors that exacerbate the incidence of gastric ulcer.

The ideal way of restoring the balance between the proteolytic capacity of the stomach (which is determined by its secretion of hydrochloric acid, pepsin and other digestive enzymes) and the protective capacity of the mucin layer is to induce the stomach to secrete mucus at a rate sufficient to coat the lining during the critical digestive periods. On the other hand, continuous replenishment of gastric acid is essential for maintaining optimal gastric function. Zinc is critical for hydrochloric acid production and gastric ulcer healing^8^. Red meats such as beef, lamb, crabmeat, lobster and salmon are rich in zinc, but unfortunately processing and overcooking reduce the bioavailability of zinc and other vital elements in these foods. Therefore, people with certain dietary habits may benefit from zinc supplementation as a way of maintaining balanced gastric activity. The investigation presented herein was conducted to evaluate the gastro-protective effect of the synthetic complex Zn(L)SCN *in vitro* against ethanol toxicity in the normal gastric cell line GES-1 and *in vivo* against ethanol-induced gastric injury in rats.

## Results

### 2-morpholino-*N*-[1-(2-pyridyl)-ethylidene] ethanamine-k3*N*,*N*′,*N*″ bis (thiocyanato-k*N*) zin(II) [Zn(L)SCN]

The compound was synthesized by reacting 2-acetylpyridine with two molar equivalents of 4-(2-aminoethyl) morpholine in the presence of zinc as shown in Fig. 1. The resulting complex was characterized by IR, ^1^H and ^13^C NMR spectroscopy, and elemental analysis. In addition, its solid-state structure was determined by single crystal X-ray diffraction.

### Cytotoxic effects of Zn(L)SCN and ethanol on the GES-1 cell line

The cytotoxicity tests indicated that the IC_50_ of Zn(L)SCN was <200 μg/mL, as shown in Fig. 2. At concentrations of 1, 5, 10, 50 and 100 μg/mL, the complex’s effects did not differ significantly from those of the vehicle (SDW). To determine whether the observed cytotoxicity was due to the compound or the ethanol solvent, we incubated the cells with different doses of EtOH (0.5, 1 and 5%) for 24 h. The tested doses significantly reduced cell viability compared to the vehicle (RPMI-1640), and the IC_50_ of EtOH was estimated to be around 1% based on the results presented in Fig. 3.

### Zn(L)SCN protected stomach cells from oxidative stress *in vitro*

Zn(L)SCN changed the level of malondialdehyde (MDA) and the activity of the endogenous enzyme SOD as shown in Fig. 4. Zn(L)SCN-treated cells exhibited significantly lower MDA levels than those treated with EtOH alone. On the other hand, the Zn(L)SCN-treated cells exhibited significantly enhanced SOD activity compared to those treated with EtOH alone. These results were very similar to those obtained for the OMP-treated cells, whose MDA levels and SOD activity were 12.28 ± 0.79 nmol/mL and 22.26 ± 0.76 U/mL, respectively. Based on these results and the viability assays (see Fig. 5), Zn(L)SCN appears to exhibit comparable protective activity to OMP. Overall, these findings indicate that Zn(L)SCN has anti-oxidant action and chemopreventive effect. To explore its action in more detail, we conducted *in vivo* studies.

### Zn(L)SCN treatment induced no symptoms of toxicity *in vivo*

Rats treated with Zn(L)SCN exhibited no evidence of toxicity over a period of 14 days. In addition, no histological changes in their hepatic or renal architecture was observed (Fig. 6), and biochemical analyses of blood samples yielded normal results, as presented in Tables 1 and 2.

### Zn(L)SCN elevated the acidity of the gastric juices and GWM, and reduced the ulcer area

In experimental animals pretreated with OMP, Zn(L)SCN at 20, 40 and 80 mg/kg, the pH of the gastric contents increased significantly compared to the control group. Low doses of Zn(L)SCN (10 mg/kg) did not imply the same increase in pH level (Fig. 7). The impact of Zn(L)SCN on gastric acidity was dose-dependent.

The effect of Zn(L)SCN on the ulcer area induced by HCl/Ethanol is shown in Fig. 8. The ulcer areas seen in the rats treated with Zn(L)SCN were significantly lower (*P* < 0.05) than those in the ulcer group, with the highest dose group (80 mg/kg) having a limited ulcer area. The rats treated with the lowest Zn(L)SCN dose (10 mg/kg) did not show any significant change in the ulcer area compared to the ulcer group. The sizes of the ulcer areas decreased as the dosage of Zn(L)SCN increased (Fig. 8).

In contrast, treatment with HCl/EtOH significantly reduced (*P* < 0.05) the mucus content of the stomach wall in the ulcer group (Alcian blue/g tissue) in comparison to the normal group (Fig. 8). The collapsed gastric mucus content was significantly (*P* < 0.05) restored in the Zn(L)SCN pre-treated animals. The highest dose of Zn(L)SCN given to the animals (80 mg/kg) resulted in a high GWM level comparable to that seen for the OMP-treated animals. The GWM level measured for the group treated with the lowest dose of Zn(L)SCN (10 mg/kg) was not significantly improved compared to the ulcer group.

### Zn(L)SCN altered gastric MDA, PGE_2_, and NO levels as well as SOD and CAT activity

The effect of Zn(L)SCN treatment on MDA levels and the activity of endogenous antioxidant enzymes SOD and CAT are recorded in Table 3. HCl/EtOH administration significantly (*P* < 0.05) elevated the level of lipid peroxidation in the ulcer group (HCl/EtOH) compared to the normal group, as indicated by the high level of gastric MDA. The different doses of Zn(L)SCN given to the animals strongly reduced the level of MDA compared to the ulcer control group, in the same way as seen for the OMP-treated groups. On the other hand, the reduced activities of SOD and CAT enzymes due to the HCl/EtOH insult were reversibly changed in the Zn(L)SCN-treated rats. The low dose of Zn(L)SCN (10 mg/kg) didn’t show significance difference in both cases.

The changes in gastric PGE_2_ levels induced by Zn(L)SCN pre-treatment are recorded in Table 3. The PGE_2_ levels in the HCl/EtOH-treated rats were significantly lower than those in the normal controls. Zn(L)SCN treatment prior to HCl/EtOH induction significantly increased PGE_2_ levels in the rats’ stomachs in a dose-dependent manner for all treatments other than the lowest dose of Zn(L)SCN (10 mg/kg), which provided no significant improvement over the HCl/EtOH-treated group. The PGE_2_ levels induced by the highest doses of Zn(L)SCN (40 and 80 mg/kg) did not differ significantly from those induced by OMP treatment, indicating that both chemicals have similar effects on the gastric tissue.

Based on the results plotted in Fig. 9, the gastric NO level was considerably lower in the stomachs of rats treated with HCl/EtOH alone compared to the normal group. Pre-treatment with Zn(L)SCN at 20, 40 or 80 mg/kg elevated the level of NO in the gastric tissue gradually, up to 39.82 ± 1.82 μM/g tissue. Once again, the results for the groups dosed with Zn(L)SCN at 40 and 80 mg/kg did not differ significantly from those for OMP-treated rats, demonstrating the potent gastroprotective effect of Zn(L)SCN.

### Zn(L)SCN attenuated the serum level of biomarkers like MPO, IL-6, TNF-α and caspase-3

The level of MPO in the serum samples collected from the ulcerated group of animals treated with only HCl/EtOH was significantly higher than for normal rats as shown in Fig. 10. The low dose (10 mg/kg), medium dose (20 mg/kg) and high doses (40 and 80 mg/kg) of the Zn(L)SCN remarkably attenuated the rats’ sera level of MPO when orally administrated one hour before HCl/EtOH treatment, depending on the dose given. Further, the serum levels observed for the medium- and high-dosage Zn(L)SCN groups were not significantly different to those for the OMP-treated group.

Data showing the effect of Zn(L)SCN on the levels of the cytokines IL-6 and TNF-α as well as the apoptotic mediator caspase-3 are presented in Table 4. The biomarker concentrations in the serum collected from ulcer rats treated with HCl/EtOH were significantly higher than those for all other groups. Conversely, rats pre-treated with different doses of Zn(L)SCN had lower values with the exception of the high caspase-3 level measured in the serum of animals treated with lowest dose of Zn(L)SCN (10 mg/kg). The serum levels seen for the rats treated with the highest Zn(L)SCN doses (40 and 80 mg/kg) were similar to those for OMP-treated animals.

### Zn(L)SCN reduced the size of ulcer lesions and the extent of neutrophil infiltration

Images of tissue sections stained with haematoxylin and eosin (H&E), and PAS are shown in Fig. 11 (I & II respectively). Gastric lesions induced by HCl/EtOH showed significant damage of the gastric mucosal epithelium. In addition, the deep lesions (black arrow) revealed obvious necrosis of the mucosa together with extensive edema (blue arrow) and submucosal infiltration of neutrophils (white arrow) into the stomach lining of the ulcer group as indicated in Fig. I b. Furthermore, PAS staining revealed depletion of gastric mucosal secretion (II b) in the same group of animals. Pre-treatment with Zn(L)SCN protected the gastric mucosa of rats as demonstrated by the reduction of ulcer lesions and neutrophil infiltration. The positive PAS staining of the mucosal lining of the stomach in the groups pre-treated with the complex indicated higher levels of mucosal glycoproteins than were present in the ulcer group (HCl/EtOH). These histological findings confirmed the biochemical results and again suggest that Zn(L)SCN has gastroprotective activity.

Images of tissue sections subjected to immunohistochemical staining for the heat shock protein Hsp70 and the apoptotic protein Bax are shown in Fig. 12 (I and II respectively). Pre-treatment of the rats with Zn(L)SCN induced over-expression of Hsp70 compared to ulcer control group animals, in which this protein was not expressed (Ib). In contrast, staining for the Bax protein demonstrated that HCl/EtOH induced injury and apoptosis in the stomachs of rats (IIb), while pre-treatment with Zn(L)SCN down-regulated Bax expression.

## Discussion

There is an urgent need for new medications with distinct physiological effects and chemically diverse structures a need, which has prompted a renewed interest in leads derived from natural sources^9^. New gastroprotective agents based on elements like zinc are usually considered less noxious, with fewer severe side effects than proton pumps and H_2_ receptor antagonists, which act by reducing hydrochloric acid production. Over 300 enzymes are currently known to be dependent on zinc for their catalytic activity^10^, and it is generally important in metabolism, growth and tissue healing^11^. Several zinc-based complexes that are ubiquitous in nature and common ingredients of human diets reportedly exhibit antiulcer activity with broad therapeutic indices. For instance, previous animal studies suggested that zinc-containing complexes and salts including zinc sulfate, meciadanol, propranolol, and dipiridamol are highly effective at treating ulcers induced by alcohol and indomethacin in rats’ stomachs. Their cytoprotective effect was attributed to changes in PGE_2_ and histamine levels in gastric mucus glands. Related zinc complexes effectively reversed changes in histamine secretion from the mucosal layer and had systematic effects on PGE_2_ production by the gastric mucosal glands^12^. *In vitro*, zinc complexes have been shown to possess antioxidant activity in cells exposed to alcohol or Non-Steroidal Anti-Inflammatory Drugs^13^; to restore serum levels of MDA, SOD and catalase (CAT); and to increase plasma antioxidant capacity^14^.

Polaprezinc (Zinc carnosine), is a patented drug that has been approved in Japan and has exhibited an efficacy of 60–70% in preclinical trials while showing a more favorable safety profile than conventional drugs. It has been shown to stop gastric ulcers in various ways, e.g. inhibiting the growth of *H. pylori*. It also reduces acid secretion and efficiently controls the corrosive effects of stomach juices, as well as having anti-inflammatory and anti-oxidant effects^15^. In addition, it increases mucosal secretion, promotes wound healing^16^, and can be used to counteract the adverse effects of NSAIDs on the stomach lining. Experimentally, zinc carnosine protected the stomach wall from mucosal erosion induced by alcohol exposure^17^ by helping to maintain adequate gastric mucus secretion. In a separate investigation, zinc carnosine treatment noticeably reduced levels of lipid peroxidation, neutrophil accumulation, and other inflammation markers in rats after aspirin-induced gastric mucosal injury^18^. In human studies, zinc carnosine treatment promoted healing within 4–8 weeks, with a higher success rate than alternative drugs^19^. The approval of Polaprezinc has prompted synthetic chemists to seek similar zinc complexes as potential improved agents for the control and treatment of gastric ulcers.

Our aim in this work was to identify zinc complexes with superior or complementary effects to those of zinc carnosine in the treatment of stomach ulcers. To this end, we investigated the gastroprotective effects of the zinc complex 2-morpholino-*N*-[1-(2-pyridyl)-ethylidene] ethanamine-k3*N*,*N*′,*N*″ bis (thiocyanato-k*N*) zin(II), or Zn(L)SCN, on acidified ethanol-induced gastric ulcers in Sprague Dawley adult rats. The organic ligand in this complex, L, is a Schiff base formed by condensing 4-(2-aminoethyl) morpholine with 2-acetylpyridine in the presence of zinc, and the analytical data for Zn(L)SCN indicate that it has a metal:ligand ratio of 1:2 20. Gastric ulcer was induced in rats by a single administration of acidified ethanol (HCl/EtOH), which were treated with Zn(L)SCN (10, 20, 40 or 80 mg/kg) one hour prior to the administration of the corrosive. The protective effect of Zn(L)SCN on the gastric lumen, was assessed by considering several variables including the activities of SOD and CAT; the levels of the prostaglandin PGE_2_ and the oxidative stress biomarkers MDA and NO; the levels of the antioxidant glutathione (GSH); the activity of the endogenous peroxides Hsp70 and Bax; and the levels of cytokines and other mediators (IL-6, TNF-α and caspase-3). The gastric mucosa and laminar gastric glands of the treated animals were subjected to histological and immunohistochemical analysis.

Our results indicated that treatment with Zn(L)SCN increased cell viability and the activity of SOD and CAT while reducing MDA levels in the HCl/EtOH-treated animals, suggesting that Zn(L)SCN exhibits protective activity against ethanol-induced oxidative stress. Oral administration of Zn(L)SCN 60 min prior to toxin ingestion improved PGE_2_ levels in a dose-dependent manner; animals treated with the highest doses of the zinc complex exhibited similar PGE_2_ levels to those seen in control rats that were not treated with HCl/EtOH. In addition, rats pre-treated with Zn(L)SCN exhibited higher levels of gastric NO than those in the ulcer group. These findings may be associated with the inhibitory effect of Zn(L)SCN on neutrophil infiltration, which was revealed by microscopic observation. Rats dosed with Zn(L)SCN prior to acid treatment also exhibited lower levels of IL-6 and TNF-α than those treated with acid alone. Histological studies indicated that Zn(L)SCN treatment resulted in intense PAS staining and a strong release of mucus, indicating efficient gastric function. Moreover, rats treated with Zn(L)SCN exhibited increased Hsp70 expression together with the downregulation of Bax and caspase-3 activity relative to ulcerated rats.

Unlike infectious diseases, gastric ulcers are multifactorial and often develop through exposure to different risk factors and unhealthy lifestyles. The mechanism of action underlying the cytoprotective activity of zinc complexes also seems to be multifaceted: our results indicate that Zn(L)SCN exhibits anti-oxidant, anti-inflammatory and anti-apoptotic activity. The pathways characterized to date suggest that zinc complexes increase the stomach’s resistance to oxidative damage induced by acute stress and reduce DNA damage and lipid peroxidation associated with apoptosis^21^. Moreover, other zinc complexes have been shown to induce the expression of Heat Shock Protein 72 (Hsp72) and inhibit that of Nuclear Factor kB (NF-kB) in the colonic mucosa, thus preventing gastric epithelial injury by inhibiting DNA fragmentation^22^. Our results showed that Zn(L)SCN promoted static and dynamic healing of gastric ulcer lesions. Moreover, it exhibited anti-apoptotic and anti-inflammatory activity, and protected against oxidative stress in a similar way to the reference drug Omeprazole, a well-known proton pump inhibitor, at doses of 40 and 80 mg/kg. We believe that its mechanism of action is based on reducing gastric acid output by suppressing neutrophil proliferation and enhancing the production of mucosal protection factors by increasing mucus secretion and microcirculation, and inhibiting H^+^ retrodiffusion. Overall, our results indicate that Zn(L)SCN treatment had positive effects on the integrity of the gastric mucosa with no side effects. Further investigations are recommended to confirm its potential as an anti-ulcer agent.

The dehydrogenase pathway is an apoptotic pathway induced by acute ethanol intoxication, which leads to the formation of excess acetaldehyde together with the generation of free radicals including secondary superoxide radicals. One of the most important mechanisms for combating oxidative stress in the intestinal microenvironment is the activation of superoxide dismutases. Ethanol ingestion leads to the accumulation of nitric oxide synthase (iNOS) and the production of the second messenger NO. Damage to the cellular membrane and enzymatic cleavage promotes overexpression of the Hsp70 and Bax genes as well as those encoding caspases, which in turn activate a set of signaling cascades. The initial step in the process is the peroxidation of lipids in the mitochondria and protein trafficking systems, leading to the formation of MDA, which is therefore widely used as a marker of oxidative stress. This process is counteracted by antioxidant enzymes such as SOD, which converts reactive oxygen species into hydrogen peroxide by superoxidation, enabling their subsequent deactivation by glutathione peroxidase and CAT. An increase in free radical production or a decrease in antioxidant activity can cause oxidative stress, which may contribute to mitochondrial damage. This in turn leads to the production of proinflammatory cytokines, followed by that of the zinc-dependent transcription factor NF-kB, which can impair the functioning of the gastric lining and thus contribute to ulcer formation. Zn(L)SCN halted the progression of gastric ulcer by downregulating IL-6 and TNF-α. Cytokine activation also has effects on downstream components with important cytoprotective effects. For example, prostaglandins are essential in the defensive mechanisms of gastric mucosa, and their production seems to be related to its free-radical-neutralizing capacity and antioxidant potential following insult with HCl/EtOH. In this work, treatment with Zn(L)SCN was shown to significantly reduce MDA levels and increase the activity of SOD and CAT while also upregulating Hsp70 and downregulating Bax and caspase 3. All of these results are consistent with a suppression of lipid peroxidation Zn(L)SCN treatment thus obstructs the inflammatory process and downregulates the inflammatory response.

Clinical perspectives

- Modern sedentary lifestyles and habits such as smoking, coffee consumption, eating fast food, and stress have been linked to digestive system malfunctions.
- A new zinc complex, Zn(L)SCN, exhibited significant protective effects against oxidative stress in addition to its anti-inflammatory and anti-apoptotic activities.
- Zn(L)SCN also exhibited gastroprotective effects against acidified ethanol-induced gastric ulcer in rats, suggesting that it may be a promising anti-ulcer therapy.

In conclusion, Zn(L)SCN effectively protected the gastric mucosa against acidified ethanol-induced injury. The mechanism of its gastroprotective activity seems to derive from its capacity to mitigate oxidative stress.

### Methods

A MEL-TEMP II instrument, a Perkin-Elmer 2400 elemental analyzer and a Bruker APEX 400 MHz FT-NMR (^1^H: 400 MHz and ^13^C: 100.4 MHz) spectrometer were used to determine melting points, conduct microanalyses, and acquire ^1^H-NMR and ^13^C-NMR spectra, respectively.

### Synthesis of 2-morpholino-*N*-[1-(2-pyridyl)-ethylidene] ethanamine-k3*N*,*N*′,*N*″ bis (thiocyanato-k*N*) zin(II) [Zn(L)SCN]

The complex Zn(L)SCN (Fig. 1) was prepared using a variant of the previously reported protocol^20^. 2-acetylpyridine (0.20 g, 1.65 mmol) and an equimolar quantity of 4-(2-aminoethyl) morpholine were dissolved in ethanol (20 mL) and heated under reflux for 2 hr, after which an aqueous solution of zinc (II) acetate dihydrate (0.36 g, 1.65 mmol) and sodium thiocyanate (0.134 g, 1.65 mmol) in water was added. The reaction was then left to stand for one hour leading to the formation of a yellowish precipitate, which was recrystallized to obtain X-ray quality crystals.

### Cell culture and cytotoxicity of Zn(L)SCN

The human gastric epithelial cell line GES-1 was originally obtained from the Chinese Academy of Sciences (Shanghai, China)^23^. The cells were cultured in RPMI-1640 medium containing 10% FBS and 1% (v/v) penicillin-streptomycin, and maintained at 37 °C under 5% CO_2_ in an incubator (NuAire Inc., Plymouth, USA).

Cell viability assays (MTT tests) were performed using the complex at various concentrations (1, 5, 10, 50, 100, 200 and 500 μg/mL) while the vehicle was left untreated. Cells were seeded at a density of 3000 cells/well with 10 μL of each treatment solution^24^. MTT solution (5 mg/mL) was then added and the cells were incubated for 3 h, after which their absorbance was recorded at 570 nm using an ELISA microplate reader (UV 1601 spectrophotometer, Shimadzu, Kyoto, Japan). The test was performed in triplicate and the results were recorded in terms of % cell viability, using equation 1:



Determination of the IC_50_ dose and the evaluation of the protective activity of Zn(L)SCN in ethanol-induced oxidative stress.

Ethanol (EtOH) is known for its ability to induce oxidative stress *in vivo* and *in vitro* models^25^,^26^. To determine the concentration of ethanol that induces 50% mortality in gastric cells, (IC_50_), GES-1 cells were cultured as described above^26^. After incubation, the cells were treated with 10 μL of SDW or an aqueous ethanol solution at one of three concentrations (0.5, 1 or 5% v/v) and the % cell viability was determined by the MTT assay.

To investigate the effects of Zn(L)SCN on ethanol-induced gastric cell mortality, four separate groups of cultured GES-1 cells were treated with SDW; the second group with 1% ethanol; the third group with 1% ethanol + Omeprazole (OMP) at a concentration of 0.04 mg/mL^27^, and the fourth group with 1% ethanol + Zn(L)SCN at a concentration of 100 μg/mL. Levels of the lipid peroxidation marker MDA were measured together with endogenous SOD activity^28^.

The level of malondialdehyde resulting from ethanol-induced oxidative stress in GES-1 cell lysates was determined colorimetrically by the Thiobarbituric Acid Reactive Substances (TBARS) assay (Cayman, USA) according to the manufacturer’s instructions. Specifically, the lysates’ absorbance at 532 nm was measured and the MDA concentration in nmol/mL was then calculated from a standard curve. SOD activity was assessed with a kit that uses tetrazolium salts to detect superoxide radicals, O_2_^−^, generated by the action of xanthine oxidase on hypoxanthine (Cayman, USA). The assays were performed according to the manufacturer’s instructions, and the SOD concentration in U/mL was calculated by measuring the lysates’ absorbance at 450 nm and comparing the result to a standard curve.

### *In vivo* experiments and acute toxicity testing

*Sprague Dawley* female rats (180–200 g weight) were used for the acute toxicity study and seven groups of 6 *Sprague Dawley* male rats (225–250 g) were used in the gastro-protective study. The rats were cared for in the animal house of the Faculty of Medicine, University of Malaya, Kuala Lumpur. All experimental protocols were carried out in accordance with the ethical guidelines and approved by the National Ethics Committee (Ethic No. PM/27/07/2012/MAA (R)) and following the criteria specified in the “Guide for the Care and Use of Laboratory Animals”.

To identify the maximum safe dosage of the complex, eighteen female rats were randomly allocated into 3 groups: a vehicle group treated with a 0.5% w/v solution of CMC at 5 mL/kg as well as low- and high-dose groups treated with Zn(L)SCN solutions at 50 and 500 mg/kg (in both cases, the animals were injected with 5 mL of treatment solution per kg) according to OECD guidelines^29^. The animals were deprived of food overnight immediately before the administration of the treatments. The animals were examined 2, 4, 8, 24 and 48 h after the treatment for periods of 30 minutes each to evaluate their clinical and toxicological status. The treated animals were kept for a period of 2 weeks and then anaesthetized with ketamine (80 mg/kg) and xylazine (10 mg/kg) after which their blood was collected for haematological and biochemical studies *via* the cardiac puncture technique. The animals were then euthanized by injection with xylazine (50 mg/kg) and ketamine (150 mg/kg), after which their kidneys and livers were collected for histological examination.

### Ulcer model and experimental design

Omeprazole obtained from the pharmacy of University Malaya Medical Centre (UMMC) was used as a reference anti-ulcer drug. The drug was dissolved in a 0.5% w/v solution of CMC for oral gavage at a dosage of 20 mg/kg body weight (5 mL/kg) following the procedure recommended by Al-Henhena *et al*.^30^.

The experiments were conducted using a slight modification of a previously reported protocol^31^. Gastric ulcer was induced using a solution of 150 mM (HCl/absolute ethanol) 40:60 v/v. Based on OECD guideline 423, four dosages of the test compound Zn(L)SCN were investigated: 1/50, 1/25, 1/12.5 and 1/6.25 of the highest dose tested in the acute toxicity test (500 mg/kg)^29^. Sixty minutes after pre-treatment, CMC was given to the normal control animals (Normal 0.5% CMC) group and HCl/ethanol (0.5%, 5 mL/kg) to the ulcer group, reference group and experimental groups in order to initiate gastric injury. The animals of the OMP reference group received an oral 20 mg/kg dose of Omeprazole while the experimental groups received Zn(L)SCN doses of 10, 20, 40 and 80 mg/kg. After an additional hour the rats were euthanized as described above with immediate excision of their stomachs.

### Gastric acidity (pH), gastric wall mucus (GWM) assessment and area measurement of gastric lesions

The pH of the gastric contents was determined by metric titration using a 0.1 N NaOH solution with a digital pH meter^32^. To assess their GWM contents, the glandular parts of the rats’ stomachs were removed and weighed^33^. A sucrose solution containing 1% Alcian blue and buffered with sodium acetate at pH 5 was used in the assays. The resulting emulsion was centrifuged and the aqueous layer’s absorbance at 580 nm was measured. The quantity of gastric wall mucus amount was estimated.

Damage to the gastric mucosa was examined to identify hemorrhagic lesions situated parallel to the stomach axis. A planimeter was used in conjunction with a dissecting microscope (1.8×) to measure the width and length of the induced ulcers based on a 10 × 10 mm^2^ area. The ulcer area was calculated as in equation 2 by the sum of the squares method using the formulas recommended by Hajrezaie *et al*.^34^:



### Gastric homogenate preparation and protein content determination

The stomachs of all rats were collected immediately after sacrifice and about 500 mg was cut from each stomach for the preparation of a gastric tissue homogenate^35^. Each stomach piece was homogenized using a Teflon homogenizer (Polytron, Heidolph RZR 1, Germany), after which the homogenate was centrifuged at 10,000 *g* for 15 minutes at 4 °C. The protein content of the collected samples was determined following Bradford’s procedure^36^. The absorbance was read at 595 nm and the protein content of each sample was calculated from a standard curve.

### Assessing malondialdehyde levels, gastric enzyme activity and nitric oxide levels in the gastric tissue

To estimate the degree of lipid peroxidation caused by the acidified ethanol (HCl/EtOH), the MDA contents of the stomach tissue homogenates were determined by means of the thiobarbituric acid (TBARS) assay, which was conducted according to the protocol outlined in the manual of the Cayman kit (Sigma, USA), in the section on *in vitro* assessment. MDA is a marker of cellular oxidative stress^37^.

The gastric content of the endogenous enzymes superoxide dismutase (SOD) and CAT were assayed according to the procedures supplied with the Cayman kits (Sigma, USA). The activity of PGE_2_ collected from the gastric tissue was assessed using 96-well microplates pre-coated with a monoclonal antibody specific to PGE_2_ according to the instructions supplied with the immunosorbent assay kit (Uscn Life Science, USA).

NO levels in the stomachs were determined by homogenizing 1 g of stomach tissue. The supernatant was collected and assayed using Griess’ reagent according to the protocol provided with the Cayman kits (Cayman, USA). The nitrate ± nitrite concentration in the gastric tissues was quantitated in units of μM/g tissue based on a nitrate standard curve plotted at 540 nm.

### Assessment of Serum Myeloperoxidase (MPO), IL-6, TNF-α and caspase-3

At the time of sacrifice, blood was collected. The serum level of MPO (indicator for neutrophil infiltration)^38^ was assayed based on the method supplied with the sandwich enzyme immunoassay kit (USCN Life Science cat. #SEA601Ra, China)^39^. In short, a microtiter plate pre-coated with an MPO-specific rat antibody was used to add standards/samples followed by the addition of Avidin conjugated to Horseradish peroxidase (HRP). The reaction was stopped with sulphuric acid and read spectrophotometrically at 450 nm.

The sera samples prepared from all animals were assayed for their levels of the inflammatory cytokines interlukin 6 (IL-6) and TNF-α as well as the apoptotic mediator caspase-3 using immunoassay ELISA kits (Uscn Life Science, cat #SEA079Ra, SEA133Ra and SEA626Ra respectively, China)^40^,^41^. The concentrations of the target antigens in the samples were determined using a standard curve equation 3 generated by analyzing standard mixtures with concentrations of 100-1.56 pg/mL for IL-6, 1000-15.6 pg/mL for TNF-α and 50-0.781 ng/mL for caspase-3.

### Microscopic evaluation of Gastric Lesions and Immunohistochemistry

Stomach specimens containing the glandular portion were fixed in 10% phosphate buffered formalin and then processed in paraffin (Leica, Germany). After processing, two types of tissue sections were prepared, both in 5 μm sections: glass microscope slides for histology and poly-L-lysine coated slides for immunohistochemistry staining. Histology slides were divided into two groups: one stained with hematoxylin and eosin for evaluation of stomach tissue histology^12^, and the other stained with Periodic Acid Schiff (PAS) stain to study the mucosal wall glycoproteins, assess mucus production, and evaluate changes in the protonation of the glycoproteins^42^.

Xylene and graded alcohol were used to deparaffinize and rehydrate the tissue sections prepared for immunohistochemistry, respectively. According to the manufacturer’s protocol (Dakocytomation, USA); the slides were prepared for immunohistochemical analysis. In brief, hydrogen peroxide (0.03%) mixed with sodium azide was used as blocking reagent for the endogenous peroxidase. After washing, the sections were incubated with Hsp70 (1:75) (Abcam cat #ab2787, USA) or Bax (1:50) (Abcam cat #ab7977, USA) biotinylated primary antibodies. The tissue sections were rinsed, placed in buffer bath and kept in a humidified chamber. A sufficient quantity of streptavidin-HRP was then added to the sections, after which they were re-incubated for 15 min followed by thorough washing. The sections were incubated for 5 min with DAB-substrate-chromagen. The sections were then washed and counterstained with hematoxylin for 5 sec followed by weak ammonia (0.037 M/L) 10 times before final mounting. Positive staining produced a brown color that was visible under the light microscope.

## Additional Information

**How to cite this article**: Salama, S. M. *et al*. A Zinc Morpholine Complex Prevents HCl/Ethanol-Induced Gastric Ulcers in a Rat Model. *Sci. Rep.* **6**, 29646; doi: 10.1038/srep29646 (2016).

## Figures and Tables

**Figure 1:** Structure of the Zn(L)SCN complex.

**Figure 2:** Cytotoxicity data for Zn(L)SCN in the normal human gastric cell line GES-1. Data are reported as Mean ± SEM (n = 3). Asterisks (*) indicate significant (*P* < 0.05) differences relative to the vehicle (RPMI-1640). SDW denotes sterile distilled water and Zn(L)SCN denotes 2-morpholino-*N*-[1-(2-pyridyl)-ethylidene] ethanamine-k3*N*,*N*′,*N*″ bis (thiocyanato-k*N*) zin(II).

**Figure 3:** IC_50_ of ethanol (EtOH). Data are reported as Mean ± SEM (n = 3). Asterisks (*) indicate significant (*P* < 0.05) differences relative to the vehicle (RPMI-1640).

**Figure 4:** Effect of Zn(L)SCN on malondialdehyde (MDA) levels and the activity of superoxide dismutase (SOD) in the human gastric cell line GES-1 under ethanol-induced oxidative stress. Data are reported as Mean ± SEM (n =3), *P < 0.05 *vs* EtOH and **P < 0.05 *vs* vehicle. (SDW) Sterile distilled water; (EtOH) ethanol; (OMP) omeprazole and (Zn(L)SCN) 2-morpholino-*N*-[1-(2-pyridyl)-ethylidene] ethanamine-k3*N*,*N*′,*N*″ bis (thiocyanato-k*N*) zin(II) [Zn(L)SCN].

**Figure 5:** Effect of Zn(L)SCN on % cell viability in the human gastric cell line GES-1 under ethanol-induced oxidative stress. Data are reported as Mean ± SEM (n = 3), *P < 0.05 *vs* EtOH and **P < 0.05 *vs* vehicle. (SDW) Sterile distilled water; (EtOH) Ethanol; (OMP) omeprazole and (Zn(L)SCN) 2-morpholino-*N*-[1-(2-pyridyl)-ethylidene] ethanamine-k3*N*,*N*′,*N*″ bis (thiocyanato-k*N*) zin(II) [Zn(L)SCN].

**Figure 6:** Acute toxicity data for Zn(L)SCN based on histological studies on kidney and liver sections of a vehicle rat treated with a 0.5% w/v solution of CMC (images (**a**,**b**), respectively), a rat treated with Zn(L)SCN at 50 mg/kg ((**c**,**d**), respectively), and a rat treated with Zn(L)SCN at 500 mg/kg ((**e**,**f**), respectively). The architecture of the kidney and liver tissue is normal in all cases. (Magnification = 20x).

**Figure 7:** Effect of Zn(L)SCN on the gastric pH for the rats from all of the experimental groups. Data are presented in the form of Mean (n = 6) ± SEM. *P < 0.001 *vs* ulcer control HCl/EtOH. **P < 0.001 *vs* normal. (CMC) Carboxymethyl cellulose; (HCl/EtOH) acidified ethanol; (OMP) omeprazole and (Zn(L)SCN) 2-morpholino-*N*-[1-(2-pyridyl)-ethylidene] ethanamine-k3*N*,*N*′,*N*″ bis (thiocyanato-k*N*) zin(II) [Zn(L)SCN].

**Figure 8:** Effect of Zn(L)SCN on the gastric wall mucus (GWM), gastric ulcer area and inhibition area % for rats from all the experimental groups. All values are displayed as Mean (n = 6) ± SEM. *P < 0.05 *vs* ulcer control HCl/EtOH. **P < 0.05 *vs* normal. ^#^*P* < 0.05 *vs* OMP-treated group. Gastric lesions’ inhibition % is recorded above the bars. (CMC) Carboxymethyl cellulose; (HCl/EtOH) acidified ethanol; (OMP) omeprazole and (Zn(L)SCN) 2-morpholino-*N*-[1-(2-pyridyl)-ethylidene] ethanamine-k3*N*,*N*′,*N*″ bis (thiocyanato-k*N*) zin(II) [Zn(L)SCN].

**Figure 9:** Effect of Zn(L)SCN on the gastric level of Nitric oxide (NO) for all treatment groups. Values are displayed as Mean (n = 6) ± SEM. *P < 0.05 *vs* ulcer control HCl/EtOH. **P < 0.05 *vs* normal control. ^#^*P* < 0.05 *vs* OMP-treated group. (CMC) Carboxymethyl cellulose; (HCl/EtOH) acidified ethanol; (OMP) omeprazole and (Zn(L)SCN) 2-morpholino-*N*-[1-(2-pyridyl)-ethylidene] ethanamine-k3*N*,*N*′,*N*″ bis (thiocyanato-k*N*) zin(II) [Zn(L)SCN].

**Figure 10:** Effect of Zn(L)SCN on the serum level of Myeloperoxidase (MPO) for all experimental animals. Values are displayed as Mean (n=6) ± SEM. *P < 0.05 *vs* ulcer control HCl/EtOH. **P < 0.05 *vs* normal control. ^#^*P* < 0.05 *vs* OMP-treated group. (CMC) Carboxymethyl cellulose; (HCl/EtOH) acidified ethanol; (OMP) omeprazole and (Zn(L)SCN) 2-morpholino-*N*-[1-(2-pyridyl)-ethylidene] ethanamine-k3*N*,*N*′,*N*″ bis (thiocyanato-k*N*) zin(II) [Zn(L)SCN].

**Figure 11:** Histological observations of HCl/EtOH-induced gastric mucosal damage in rats (I) H&E staining. (II) PAS staining of the mucus layer. (**a**) Normal control rats showing normal gastric mucosa. (**b**) Ulcer control rats showing severe damage of the surface epithelium (black arrow), submucosal edema (blue arrow) and neutrophil infiltration (white arrow). (**c**) OMP-treated rats (20 mg/kg) showing mild gastric damage and intense mucus secretion. (**d**–**g**) Experimental rats pre-treated with Zn(L)SCN (10, 20, 40 and 80 mg/kg respectively) showing protection of the surface epithelium indicated by the decrease in mucosal damage and neutrophil infiltration, and increase in the mucus layer. (H & E stain 10x and PAS stain 20x).

**Figure 12:** Effect of Zn(L)SCN on the immunohistochemical staining of Hsp70 (I) and Bax (II). (**a**) Normal stomach. (**b**) Ulcer control group animals (HCl/EtOH) showing no Hsp70 expression and over-expression of Bax (dark red arrow). (**c**) OMP-treated animals (omeprazole, 20 mg/kg) showing over-expression of Hsp70 (orange arrow) and down expression of Bax. (**d**–**g**) Rats received 10, 20, 40 and 80 mg/kg of Zn(L)SCN, respectively showing significant over-expression of Hsp70 and reduced expression of Bax protein. (Magnification = 20x).

**Table 1:** Renal function data from the acute toxicity testing of Zn(L)SCN.

Dose	Sodium (mmol/L)	Pottasium (mmol/L)	Chloride (mmol/L)	Urea (mmol/L)	Creatinine (μmol/L)
Vehicle (CMC 0.5%)	139.52 ± 1.24	4.80 ± 0.53	105.52 ± 1.36	5.50 ± 0.50	39.79 ± 2.71
Zn(L)SCN (50 mg/kg)	143.23 ± 1.98	4.90 ± 0.47	103.70 ± 2.14	5.11 ± 0.49	39.92 ± 2.19
Zn(L)SCN (500 mg/kg)	139.89 ± 2.55	5.16 ± 0.26	104.68 ± 0.95	5.28 ± 0.49	39.10 ± 3.00

Data are recorded as Mean ± SEM (n = 6). No significance (*P* > 0.05) was marked between the tested groups.

**Table 2:** Liver function data from the acute toxicity testing of Zn(L)SCN.

Dose	Total protein g/L	Albumin (g/L)	Globulin (g/L)	TB (μmol/L)	AP (IU/L)	ALT (IU/L)	AST (IU/L)	GGT (IU/L)
Vehicle (CMC 0.5%)	68.00 ± 1.67	11.77 ± 0.73	56.10 ± 0.91	1.83 ± 0.15	69.84 ± 4.66	37.83 ± 2.39	166.32 ± 1.86	4.42 ± 0.20
Zn(L)SCN (50 mg/kg)	70.97 ± 1.26	12.56 ± 0.50	58.39 ± 0.70	2.16 ± 0.10	64.52 ± 4.59	39.14 ± 3.15	168.41 ± 1.82	4.70 ± 0.43
Zn(L)SCN (500 mg/kg)	68.86 ± 1.84	12.87 ± 0.32	57.44 ± 1.32	1.97 ± 0.13	79.40 ± 4.60	34.48 ± 2.91	167.68 ± 1.55	4.72 ± 0.31

Data are recorded as Mean ± SEM (n = 6). No significance (*P* > 0.05) was marked between the tested groups.

**Table 3:** The effect of Zn(L)SCN on MDA levels and the activity of SOD, CAT and PGE_2_ in the gastric tissue from all experimental rats.

Group	MDA (nmol/mg protein)	SOD (U/mg protein)	CAT (nmol/min/mg protein)	PGE_2_ (pg/mg protein)
Normal (CMC 0.5%)	13.33 ± 0.92	50.50 ± 1.79	36.24 ± 1.13	342.35 ± 9.10
HCl/EtOH	77.94 ± 4.96**	17.96 ± 1.21**	15.86 ± 1.86**	110.76 ± 3.59**
OMP 20 mg/kg	16.70 ± 1.18*	46.44 ± 2.38*	37.20 ± 2.22*	327.12 ± 3.72*
Zn(L)SCN 10 mg/kg	61.88 ± 6.47*,#	23.69 ± 1.99#	23.31 ± 1.60*,#	119.37 ± 4.81#
Zn(L)SCN 20 mg/kg	31.90 ± 2.76*	33.67 ± 2.59*,#	26.28 ± 1.43*,#	226.58 ± 4.59*,#
Zn(L)SCN 40 mg/kg	21.59 ± 2.14*	45.16 ± 1.91*	38.72 ± 0.97*	303.13 ± 6.06*
Zn(L)SCN 80 mg/kg	16.11 ± 1.66*	51.78 ± 2.23*	41.02 ± 1.11*	319.96 ± 5.34*

Data are presented in the form of Mean ± SEM (n = 6).

*P < 0.05 *vs* ulcer control HCl/EtOH.

**P < 0.05 *vs* normal control.

^#^*P* < 0.05 *vs* OMP-treated group. (MDA) Malondialdehyde; (SOD) superoxide dismutase; (CAT) catalase; (PGE_2_) Prostaglandin E_2_; (CMC) carboxymethylcellulose; (HCl/EtOH) acidified ethanol; (OMP) omeprazole and (Zn(L)SCN) 2-morpholino-*N*-[1-(2-pyridyl)-ethylidene] ethanamine-k3*N*,*N*′,*N*″ bis (thiocyanato-k*N*) zin(II) [Zn(L)SCN].

**Table 4:** The effect of Zn(L)SCN on the level of IL-6, TNF-α and caspase-3 in the serum from all experimental rats.

Group	IL-6 (pg/mL)	TNF-α (pg/mL)	Caspase-3 (ng/mL)
Normal (CMC 0.5%)	1.74 ± 0.06	14.87 ± 1.25	2.71 ± 0.27
HCl/EtOH	13.42 ± 0.53**	108.80 ± 4.88**	18.88 ± 2.21**
OMP 20 mg/kg	1.86 ± 0.08*	18.95 ± 1.99*	2.58 ± 0.23*
Zn(L)SCN 10 mg/kg	5.39 ± 0.46*,#	70.76 ± 3.43*#	14.19 ± 1.71#
Zn(L)SCN 20 mg/kg	4.22 ± 0.17*,#	52.85 ± 3.10*,#	5.66 ± 0.43*
Zn(L)SCN 40 mg/kg	2.74 ± 0.15*	21.57 ± 1.27*	2.01 ± 0.19*
Zn(L)SCN 80 mg/kg	2.31 ± 0.07*	17.34 ± 0.69*	2.32 ± 0.20*

Data are presented in the form of Mean ± SEM (n = 6).

*P < 0.05 *vs* ulcer control HCl/EtOH.

**P < 0.05 *vs* normal control.

^#^*P* < 0.05 *vs* OMP-treated group. (IL-6) Interlukin-6; (TNF-α) Tumor necrosis factor-α; (CMC) Carboxymethyl cellulose; (HCl/EtOH) acidified ethanol; (OMP) omeprazole and (Zn(L)SCN) 2-morpholino-*N*-[1-(2-pyridyl)-ethylidene] ethanamine-k3*N*,*N*′,*N*″ bis (thiocyanato-k*N*) zin(II) [Zn(L)SCN].
